This article has been retracted.

# Construction and optimization of inventory management system via cloud-edge collaborative computing in supply chain environment in the Internet of Things era

**DOI:** 10.1371/journal.pone.0259284

**Published:** 2021-11-03

**Authors:** Hailan Ran

**Affiliations:** Xi’an Fanyi University, Xi’an City, China; Ministry of Natural Resources North Sea Bureau, CHINA

## Abstract

The present work aims to strengthen the core competitiveness of industrial enterprises in the supply chain environment, and enhance the efficiency of inventory management and the utilization rate of inventory resources. First, an analysis is performed on the supply and demand relationship between suppliers and manufacturers in the supply chain environment and the production mode of intelligent plant based on cloud manufacturing. It is found that the efficient management of spare parts inventory can effectively reduce costs and improve service levels. On this basis, different prediction methods are proposed for different data types of spare parts demand, which are all verified. Finally, the inventory management system based on cloud-edge collaborative computing is constructed, and the genetic algorithm is selected as a comparison to validate the performance of the system reported here. The experimental results indicate that prediction method based on weighted summation of eigenvalues and fitting proposed here has the smallest error and the best fitting effect in the demand prediction of machine spare parts, and the minimum error after fitting is only 2.2%. Besides, the spare parts demand prediction method can well complete the prediction in the face of three different types of time series of spare parts demand data, and the relative error of prediction is maintained at about 10%. This prediction system can meet the basic requirements of spare parts demand prediction and achieve higher prediction accuracy than the periodic prediction method. Moreover, the inventory management system based on cloud-edge collaborative computing has shorter processing time, higher efficiency, better stability, and better overall performance than genetic algorithm. The research results provide reference and ideas for the application of edge computing in inventory management, which have certain reference significance and application value.

## Introduction

With the rapid development of science and technology, the combination of manufacturing processes, industrial IoT (Internet of Things), advanced computing, and other technologies has become increasingly close. Meanwhile, the manufacturing mode has changed from a product-centric mode to a user-centric mode [1, 2]. Due to the complexity of business processes in large manufacturing plants, it is necessary to coordinate the relationship between people, information system, and physical system, which causes the traditional imbalance between resource allocation and task planning [3]. Moreover, concepts such as the intelligent plant, intelligent transportation and smart city have emerged as AI (artificial intelligence) and computer technology develop fast. Lv et al. (2018) designed a new government service platform by using 3D (three-dimensional) geographic information system and cloud computing to effectively manage and use urban data. In addition, they achieved the 3D analysis and visualization of urban information through the smart city platform, which made the life of the masses more convenient [4]. This proves that the application of computer and AI technology has become a hot research topic.

The development of China’s industry in the next decade will shift from labor-intensive production to technology-intensive production, which will bring great progress in advanced technology. Correspondingly, domestic enterprises have begun to explore the transformation approach to adapt to market changes and meet government needs. The fast-growing IoT applications can produce enormous amounts of data at the network edge, effectively promoting the generation and development of edge computing. Edge computing is one of the crucial technologies to realize intelligent industry. In large manufacturing workshops, sensors, instruments, and intelligent devices can collect mass of machine data [5]. These kinds of data are the main sources of industrial big data. Moreover, it is difficult to effectively master and forecast market demands. To reduce the dependence on the accuracy of market demand forecasting and improve the efficiency of supply chain inventory management, it is necessary to improve inventory management efficiency to adapt to the changes in market demand. Besides, it is essential to use management methods to compensate for many negative impacts of market uncertainty [6]. In this case, the upstream and downstream enterprises of the supply chain must create a constant speed supply chain based on the network platform to reduce the inventory cost of the supply chain and meet the needs of customers in real time. Industrial big data is considered as a necessary means to further enlarge product profit margin. At present, industrial data platform is the paramount component of data storage, calculation and analysis for intelligent factories. With the increase in smart devices in smart factories, a large number of data such as RFID (radio frequency identification) is obtained, providing a rich data set for the manufacturing industry. As IoT applications develop rapidly, mass of data is generated at the edge of the network, effectively facilitating the emergence and development of edge computing. Consequently, in large manufacturing workshops, sensors, instruments, intelligent terminals, and other devices can collect a large amount of machine data, as the main source of industrial big data. Under the background of increasingly socialized mass production and global economic integration, all links of the supply chain, such as raw material supply, production, logistics, consumption, processing, distribution, and retail must cooperate closely. Nevertheless, the coordination and management in all links, including inventory management, are still relatively closed, significantly reducing the comprehensive benefits of the overall supply chain.

The industrial production data is investigated here based on the analysis of the related concepts and production modes of supply chain and cloud manufacturing. Then, the demand prediction method for different types of industrial spare parts and the inventory management system are proposed via cloud-edge collaborative computing. The purpose of this work is to optimize inventory management and utilization efficiency by predicting the demand for vulnerable spare parts, and improve the performance of inventory management system with the advantage of cloud-edge collaboration computing. Moreover, cloud computing and IoT technology are utilized to explore the implementation method of refining the traditional inventory management of the supply chain. The innovation of this study is that corresponding demand prediction methods are studied separately according to three demand modes of vulnerable spare parts, namely periodic demand, stationary demand, and trend demand. Specifically, the simple exponential smoothing method is used to predict demand of stationary spare parts. The quadratic exponential smoothing method is selected to predict the linear demand, and the feature synthesis method is proposed for forecasting the spare parts with periodic demand mode. On this basis, edge computing is employed to develop a cloud-edge collaborative computing architecture, to optimize the spare parts prediction algorithm and improve inventory management efficiency and pertinence.

## Related theories and research methods

### Overview and status of supply chain inventory management

IoT technology is the combination of intelligent recognition technology, wireless sensor technology, ubiquitous computing technology, and network technology. The global IoT network is still in the stage of concept, demonstration, and test, many key technologies need to be further studied, and standardization norms need to be further developed. However, it has triggered the third wave of information industry development in the world after computers and the Internet, which is an impactful upgrade of the application of information technology to human production and life. Supply chain is a kind of complete and functional network chain consisting of suppliers, manufacturers, distributors, retailers and end users centering on the business center enterprise and formed through controlling feed-forward information flow and the feedback of material flow and information flow [7]. There are diversified research works about supply chain inventory management. Bornkamp (2019) emphasized the importance of supply chain in his research. The author believed that the renegotiation of the UK-EU relationship would most likely take several years, but European distributors had to assess their current inventory management to mitigate future disruptions. Moreover, with the political pattern continuing to change, the growing e-commerce market would bring trade growth, so managing availability and distribution of inventory was critical to reducing overall costs, improving cash flows and increasing flexibility in supply chain operations, in order to effectively serve the European market [8]. Aaha et al. [9] analyzed six professional education courses offered by THE Council of Supply Chain Management Professionals, including senior certified professional forecaster, certified production and inventory management professionals, certified supply management professionals, and supply chain professionals. They took personal interests and organizational interests as the two main standards, and took the professional education plan as an alternative [9]. Evidently, people have gradually realized the significance of supply chain, and delved into supply chain deeply and professionally. Fig 1 reveals the basic structure of the supply chain.

**Fig 1:** Basic structure of supply chain.

The supply chain not only aggerates the logistics information and funds of suppliers and users, but also forms its own value. In the distribution link of the supply chain, the appreciation in products has been achieved through packaging, processing, transportation, and delivery. Supply chain inventory management is the process of defining the overall goal of supply chain inventory management and reviewing the inventory strategy of enterprises on supply chain nodes. The supply chain inventory management aims to sustain the optimal overall supply chain inventory and reduce the total inventory to respond to changing market demands. The improvement of the cost of supply chain inventory and supply chain can enhance the rapid response of inventory to the market.

### Introduction to concepts related to cloud-edge collaboration for logistics management

Cloud manufacturing includes cloud-edge collaboration technology, AI service technology, container-based platform service technology, digital twins service technology, data security, and other related technologies. It is a novel type of digital, intelligent, and smart networked manufacturing with Chinese characteristics. Fig 2 reveals the overall schematic of the system of cloud manufacturing technology.

**Fig 2:** Overall system of cloud manufacturing technology.

The foundation of intelligent cloud manufacturing is a ubiquitous and human-centered network, which integrates digital technology such as information manufacturing technology and intelligent technology comprehensively [10]. The cloud manufacturing system enables users to obtain manufacturing resources and capabilities according to their own needs anytime and anywhere through the cloud-based manufacturing service platform, and intelligently perform various activities throughout the life cycle.

In the industrial field, the IoT proactively identifies and remotely controls all physical devices in the cloud manufacturing scenario of existing network infrastructure, and obtains content in the physical world (real space) in the information world (cyberspace). The data reflects the whole life cycle of the corresponding physical equipment, and realizes the digital twins [11, 12].

Internet technology facilitates the active and independent analysis of industrial product manufacturing process, generates intelligent perception and active prediction of the outside world, and forms a closed-loop process of automatic repair and complete feedback. With the emergence of intelligent control, industrial IoT can optimize all aspects of industrial systems, including intelligent manufacturing and business systems, real-time monitoring, supply chain collaboration, value-added services, and other business needs. The wide application of industrial IoT technology makes the production process more active and intelligent, which can accurately predict and effectively solve the potential obstacles, to effectively increase corporate profits [13, 14].

The continuous development of the mobile Internet has brought new convenience for people’s life and production, as well as more needs and challenges, such as higher requirement of timeliness, security, and reliability. Hence, edge computing is needed to improve cloud computing ability. Fig 3 illustrates the typical architecture of edge computing for intelligent plants.

**Fig 3:** Typical architecture of edge computing for intelligent plants.

Many problems such as single-point faults may occur in industrial applications. In addition to the unified control of the cloud, the edge nodes have the computing ability to independently make decisions and solve problems, which can improve factory productivity, while avoiding equipment failure. In IoT scenarios, edge computing focuses on solving problems of lightweight data size closer to the user’s by transferring computing operation [15]. Therefore, it cannot completely replace cloud computing, but assists cloud computing to improve work efficiency. With the deepening of industry research and academic research, cloud collaboration is widely used in numerous fields such as medical treatment, industry, and finance. Cloud-edge collaborative architecture can balance the load and reduce the hardware requirements of edge devices, making the peripheral equipment more convenient while maintaining the capacity [16, 17]. Fig 4 provides a manufacturing factory example based on cloud-edge collaborative computing architecture.

**Fig 4:** The manufacturing factory based on cloud-edge collaborative computing architecture.

### Demand prediction of vulnerable spare parts in IoT supply chain environment

In the cloud manufacturing scenario, the amount of data sent by the terminal equipment deployed in each plant is different for various plant equipment and actual business needs. Therefore, it is necessary to design a scheme for the edge server equipped in different plants to effectively reduce the procurement funds of enterprises and avoid the waste of limited resources. Based on this consideration, a demand prediction method is proposed for vulnerable spare parts, and it is combined with the cloud-edge cooperative inventory management system to improve the efficiency and quality of inventory management.

Timely maintenance and supply of spare parts are two important components of the after-sales service system provided by large equipment manufacturers in the service network [18]. Among them, the efficiency of spare parts inventory management determines whether spare parts can reach the demand in time, which directly affects the market competitiveness of service systems and manufacturers. In the IoT era, many consumption data and consumption behaviors based on IoT provide sufficient data basis for market demand prediction. Shen et al. (2020) extracted knowledge from user generated content and depicted the differences between IT service companies’ use of social media and users’ expectations based on daily interaction between suppliers with customers [19]. The data analysis method is also adopted here to forecast the spare parts demand.

The purpose of inventory management is to deal with various changes and uncertainties in spare part supply to ensure the normal operation of spare part supply. According to the function and direction of spare parts, they can be divided into two categories: maintenance spare parts and service spare parts.

The function of maintenance spare parts is to ensure the normal operation of production equipment, while the function of service spare parts is to ensure the after-sales service of products. Different types of spare parts have diverse inventory management purposes and management methods [20]. In summary, in the case of low total cost of spare parts inventory, it is very practical to study how to optimize the inventory management system according to the actual situation of enterprises to achieve a significant improvement in service level. The spare parts inventory management strategy includes spare parts classification, spare parts demand analysis, spare parts shortage management, spare parts inventory mode, and inventory strategy.

The common vulnerable parts of pump trucks in industrial production are taken as the research object here to predict their needs, including conveying cylinder, concrete piston, and cutting ring, usually with relatively large demands. Through the analysis of the sales volume of concrete piston in different regions, the demand is classified into the following three categories: periodic demand time series, demand time series with rising trend, and stable demand time series [21].

The prediction based on periodic demand time series is first discussed. Spare parts with periodic changes in demand patterns include random components and periodic components in the past demand time series [22, 23]. The proposed prediction method calculates the cycle length according to the time series of spare parts demand in the past, calculates the demand data of original spare parts according to the cycle length, and divides each segment and performs polynomial fitting. The polynomial function of each cycle is integrated to obtain a new polynomial function to extract periodic ports and remove random factors, which is used as a prediction model to predict the demand of the next period.

Generally, the demand data of a part may have a constant cycle, but the cycle means that the demand data of the cycle interval have similar fluctuations rather than being identical to each other [24, 25]. To detect the period of a time series, the most important thing is to solve the problem of accurately measuring the similarity of time series. For the similarity measurement of two time series, most studies adopt the Euclidean distance method. The smaller the distance measure is, the more similar the two time series data are. The Euclidean distance can be expressed as Eq (1).

$$d(\text{T},\text{S})=\frac{1}{n}\sqrt{\sum_{i=1}^{n}{\left(t_{i}-s_{i}\right)}^{2}}$$ (1)

In Eq (1), *T* is the target time series, *S* denotes the time series needed for similarity measurement, and *n* represents the length of two time series. Besides, *t*_*i*_ or *s*_*i*_ refers to a factor at a time in a time series.

Euclidean distance represents the proximity of distance between two time series, but does not reflect the dynamic trend. The similarity between the two data can also be proved by the fact that the overall trend of variability is consistent and uniformly correlated. Therefore, correlation coefficient can be used as another measure of similarity, which can be written as Eq (2).

$$\text{f}(\text{T},\text{S})=d(\text{T},\text{S})-p_{TS}$$ (2)

In Eq (2), *P*_*TS*_ refers to the correlation coefficient of time series. Meanwhile, *d*(*T*, *S*) stands for the Euclidean distance of two time series data, and *f*(*T*, *S*) is the similarity measure function.

Eq (3) indicates the detection of period length based on similarity.

$$F(\text{C})=\frac{2}{\left[\frac{n}{C}\right](\left[\frac{n}{C}\right]-1)}\sum_{D_{i,}D_{j}\in X_{C}}f(D_{i,}D_{j})$$ (3)

In Eq (3), *X* stands for a given time series. Besides, *D* represents a fragment in a given time series, and C denotes the time length of the fragment.

T=min{F(C)|C=a∼b,F(C)≤α} (4)

In Eq (4), the value of *a* is 1, and the value of *b* is n/2. *α* signifies the threshold.

Once the duration length period of the time series is calculated, the whole time series can be divided into multiple duration periods according to the duration length period. The analytic expression of the function for each cycle is unknown, but the data points on each cycle are known. It is essential for the extraction of the periodic function from each cycle to analyze the known cycle so that the internal data points are matched with the function. Due to the different influence of external factors on spare parts demand in each period, the time period extracted by fitting function cannot represent the periodic trend of the whole time series [26]. Therefore, the fitting functions of each period are integrated to form a new adjustment function to remove the influence of random factors, which is used as the periodic equation of all periods (time series), as shown in Eq (5).

$$p(x)=a_{k}x^{k}+a_{k-1}x^{k-1}+\ldots +a_{1}x+a_{0}$$ (5)

There are several methods to predict the continuous demand of spare parts for the non-periodic demand time series, such as the exponential smoothing method and the weighted moving average method. The exponential smoothing method is an improvement of moving average method characterized by simple form, easy implementation, and high precision, which can accurately reflect the changes in demand data and is widely used in practice. Therefore, the exponential smoothing method is selected as the spare parts demand prediction method based on aperiodic demand time series here.

When the spare part data does not follow a linear trend, the demand model of exponential smoothing prediction is presented in Eq (6).

$$m_{t+1}^{/}=am_{t}+(1-a)m_{t}^{/}$$ (6)

In Eq (6), *a* represents a smoothing constant, and $m_{t+1}^{/}$ denotes the predicted value of the (*t*+*1*) period.

When the spare parts data does not meet the linear trend, the demand model for exponential smoothing prediction needs to be smoothed twice, as shown in Eqs (7) and (8), respectively.

$$n_{t+1}^{}=an_{t}+(1-\text{a})n_{t}^{}$$ (7)

$$z_{t+1}^{/}=an_{t+1}+(1-\text{a})z_{t}^{/}$$ (8)

Among Eqs (7) and (8), *a* denotes the smooth constant, and *S*_*t*+*1*_ stands for the smooth value of (t+1) period.

For the prediction of intermittent time series, the intermittent demand time of spare parts has two characteristics. (1) There is less demand. In other words, there is no demand during this period. (2) There is great volatility in demand value. These two characteristics cause a large prediction error of intermittent time series [27]. Furthermore, the time aggregation prediction method is used to predict the demand of intermittent time series.

### Inventory management system based on cloud-edge collaboration

Core competitiveness is crucial to large equipment manufacturers, because efficient management of spare parts inventory can effectively reduce costs and improve service levels. The engineering machinery and equipment usually have a complex structure and various components and parts. However, the existing spare parts inventory management is still cumbersome and unsystematic, which determines inventory according to personal experience and plans demands according to inventory proportion, bringing great pressure to the production department and other related departments. The solution of traditional cloud computing architecture is to download the sensor data of various factory equipment, and use the data analysis technique of big data. Meanwhile, it transits the downloaded data to remote cloud servers through the data acquisition module, to improve work efficiency and competitiveness [28, 29]. Here, the cloud-edge collaborative computing in industrial IoT is proposed to solve the rapid response problem of real-time control and data fast processing in large-scale manufacturing plants. Fig 5 provides the architecture of cloud-edge collaborative computing.

**Fig 5:** Architecture of cloud-edge collaborative computing.

The deployment of industrial IoT in intelligent manufacturing environment mainly contains the equipment perception layer, data resource layer, service application layer, and operation and maintenance management layer, which work together to maintain all data links [30, 31]. From the specific business point of view, the cloud components are mainly responsible for the formation of the model of the collected data, and the peripheral components are basically responsible for obtaining the model from the data dictionary, providing timely services for factory equipment in real time. Reducing the training time of models and networks can shorten the response time of the closed-loop system and improve the overall production quality of the plant equipment. OpenStpack and Starling X enable companies to build their own cloud- edge collaborative computing services using the most advanced open-source cloud computing platform and the latest distributed cloud computing platform, respectively.

The solution of traditional cloud computing architecture is to upload all kinds of sensor data from factory equipment, such as vibration, pressure, and temperature, to the cloud remote server through data acquisition module. Besides, it utilizes the popular big data analysis technology to establish the mathematical model of index data and factory equipment performance, to enhance the production quality, work efficiency, and market competitiveness of factory equipment. Taking the coal industry as an example, the mine is generally located in a remote location where it is difficult to implement network communication. Due to the characteristics of large scale, numerous varieties, low value density, and fast update and processing requirements of coal mine data, the traditional cloud computing architecture is inadequate, because it is easy to produce problems of single point faults and slow closed-loop response. Based on the above analysis, the cloud-edge collaborative computing architecture is selected for the industrial IoT to cope with the problems of fast real-time control response and fast data calculation in large manufacturing workshops. Fig 6 illustrates the workflow of cloud-edge collaborative computing architecture, where various data acquisition devices and user requests are collectively referred to as collectors. The smart endpoint simply pre-processes information from the collectors and sends it to the computing node in the edge server cluster [32]. Then, the I/O intensive virtual machine on the computing node receives the information and stores it in the database on the storage node.

**Fig 6:** Workflow of cloud-edge collaborative computing.

The following is the specific processing of the edge server:

1. the intelligent terminal sends the collected data to the edge data storage module;
2. data processing module retrieves the corresponding data from the edge data storage module according to the user’s request;
3. data processing module carries out lightweight big data analysis according to the model parameters provided by the data dictionary module. Besides, the edge data dictionary module is analyzed and synchronized;
4. the decision module outputs the processing results of the data processing module to the intelligent equipment and checks them accordingly.

The procedure of the remote centralized server is as follows:

1. the edge server and remote centralized data storage module synchronize incremental data;
2. data processing module retrieves data from the remote centralized data storage module according to user needs;
3. the data processing module conducts large-scale big data analysis according to the model parameters provided by the data dictionary module.

The analysis and synchronization of the remote data dictionary module are presented as follows:

1. edge server synchronizes incremental data with the remote centralized data storage module;
2. the data processing module retrieves data from remote centralized data storage module according to user needs;
3. the data processing module conducts large-scale big data analysis according to the model parameters provided by the data dictionary module. Meanwhile, analysis and synchronization are performed on the remote data dictionary module;
4. the remote data dictionary module synchronizes data processing with edge data dictionary module according to specific requirements.

Edge servers and remote centralized servers regularly analyze and use stored data, and the data dictionary is updated to ensure the correctness of the decision message.

### Simulation and experimental design

Three time series prediction methods are provided for the demand prediction of vulnerable parts based on spare parts. The demand data of high-strength circular chains in the mining industry is used here for verification. The circular chain is also a spare part of construction machinery, and the experimental data comes from the network. In the simulation experiment, the genetic algorithm is introduced as a comparative algorithm to verify the performance of the inventory management system based on cloud-edge collaborative computing architecture. Table 1 indicates the task parameters under different configurations in this experiment.

**Table 1:** Setting of experimental parameters.

Task	1	2	3	4	5	6
**Type**	World Count	World Count	Sort	Sort	Tcra	Tcra
**Data set specification /MB**	108	108	216	216	432	432
**Completion time /s**	20	20	23	23	25	25

### Analysis of demand prediction results and the performance verification of inventory management system

#### Comparison results of the prediction method based on demand of vulnerable spare parts

After the prediction model is established, the predicted value of spare parts demand is calculated to be compared with the true value. The polynomial is established and fitted according to the period length. Fig 7 illustrates the relationship between fitting times and prediction errors.

**Fig 7:** Relationship between fitting times and prediction errors.

Fig 7 shows that the prediction error decreases first and then increases with the increase of fitting times. When the fitting time of the polynomial reaches 10, the prediction error begins to stabilize. After 13 times of fitting of the polynomial, the prediction error reaches a minimum of 11.7%, and then begins to increase. Based on this result, in the following simulation experiment, 13 times of fitting are used to obtain the fitting polynomial of each section when the polynomial regression model is used to fit the demand data of spare parts.

The eigenvalues and the weighted fitting process of each cycle are shown in Fig 8.

**Fig 8:** Eigenvalues and the weighted fitting processes ((a): eigenvalues of each cycle; (b): weighted fitting processes of each cycle).

Fig 8 displays the intermediate process of eigenvalue fitting. As can be seen from Fig 8B, the prediction error of monthly demand after weighted fitting is smaller. The mean value of the sum of eigenvalues and the weighted sum of eigenvalues shown in Fig 8A is used to synthesize new feature sets. In other words, the determination of values of a_n_, b_n_, and c_n_ is similar to the determination of polynomial degree. Through experimental analysis, the prediction accuracy is the highest when w = 0.1, w = 0.1, and w = 0.8.

Fig 9A illustrates the mean value of the sum of eigenvalues and the weighted sum of eigenvalues shown in Fig 8A. Fig 9 provides the prediction results of spare parts demand based on the weighted synthesized eigenvalues.

**Fig 9:** Prediction results of spare parts demand based on weighted eigenvalues ((a): weighted eigenvalues; (b): prediction results based on weighted eigenvalues; (c): error comparison of two processing methods).

According to Fig 9b, from a macro perspective, the prediction result based on the weighted sum is closer to the real value than the prediction based on the mean value of sum of the eigenvalues. From the perspective of error value, the highest prediction error based on the weighted eigenvalues is 34.9%, and the lowest is 2.2%. Through the comparison of error in Fig 9C, the average relative error based on the weighted fitting is lower than that based on the mean value of the sum of eigenvalues, the former is 11.7%, and the latter is 18.4%. Therefore, the prediction accuracy of the prediction model established by the weighted fitting method is higher. To sum up, the prediction method based on weighted fitting of eigenvalues has the smallest error and the best fitting effect in the demand prediction of machine spare parts.

**Verification results of the perdition method based on vulnerable spare parts demand.** The simulation experiment adopts the moving average period coefficient prediction of the prediction method based on weighted eigenvalues as a comparison with the true value. The specific results are presented in Fig 10.

**Fig 10:** Weighted eigenvalues and prediction results ((a): weighted eigenvalues; (b): fitting processing of weighted eigenvalues; (c): comparison between prediction results and true results).

In Fig 10A, a_n_ refers to the first set of eigenvalues, b_n_ denotes the second set of eigenvalues, c_n_ represents the eigenvalues after fitting, the value range of cycle length is 1 ~ 13, and the threshold is 10% of the mean value. Polynomial fitting is carried out for the first two data segments to obtain the periodic term of the data segment, which is used to predict the true value of the third cycle segment. When n = 10, the prediction error is the smallest, so the degree of the fitting polynomial is n = 10. The fitting polynomial function of each segment is obtained. From Fig 10, the average relative error between the actual value of spare parts demand and the predicted value is 9.4%. When the moving period coefficient method is used to predict the demand for spare parts, the average relative error between the predicted value and the actual value is 13.0%.

The proposed prediction method is also used to predict the demand of the circular chain, and the results are compared with those of the moving average period coefficient method, to further verify the advantages of this method. The comparison results are shown in Fig 11.

**Fig 11:** Comparison of the results of two prediction methods.

From Fig 11, the average absolute error of the actual value and predicted value of spare parts demand based on the moving average period coefficient method is 286.8, and the average relative error is 12.8%. The average absolute error of the polynomial fitting model is 250.7, and the average relative error is 11.7%. Therefore, the proposed prediction mode has a better prediction effect.

The prediction results of exponential smoothing method and quadratic exponential smoothing method are shown in Fig 12.

**Fig 12:** The prediction results of exponential smoothing method and quadratic exponential smoothing method ((a): the prediction results of exponential smoothing method; (b): the prediction results of quadratic exponential smoothing method).

The simple smoothing index prediction method is used to investigate the spare parts demand data with the nonlinear trend. According to Fig 12A, the predicted value of spare parts demand by smoothing index prediction method is close to the actual value, and the average relative error is 18.0%. The quadratic smoothing index prediction method is aimed at the spare parts demand data with linear trend. From the results in Fig 12B, the predicted value of demand of the quadratic exponential smoothing method is close to the actual value, and the average relative error is 11.3%. In conclusion, the exponential smoothing method and quadratic exponential smoothing method both have high prediction accuracy in spare parts demand.

To sum up, the cycle length detection method based on similarity is adopted to calculate the cycle length. Then, the data is divided into several segments according to its cycle length, and polynomials are used to fit the data in the cycle segment. Moreover, the polynomials are synthesized to obtain a new polynomial function, which is used as the prediction model to predict the demand in the next cycle. The experimental results demonstrate that this prediction method can achieve high prediction accuracy.

**Performance verification results of inventory management system based on cloud-edge collaborative computing.** The algorithm of the inventory management system optimizes the resource allocation for virtual machines from the impact of virtual machines on the performance of physical machines and the impact of different configurations of virtual machines on task execution time. Table 2 and Fig 13 signify the resource allocation scheme for the best virtual machine performance obtained by the two algorithms and the comparison of the results after 100 executions of six tasks at the same time, respectively.

**Fig 13:** Performance comparison between two algorithms ((a)-(f) represent the experimental results from Task 1 to Task 6).

**Table 2:** Allocation plan of CPU.

Parameter	CPU1	CPU2	CPU3
**Research algorithm**	5	5	6
**Genetic algorithm**	5	5	6

Fig 13 illustrates the performance comparison between the proposed algorithm and the genetic algorithm. Specifically, the average completion time of the six tasks executed by the genetic algorithm is 15.64 seconds, 14.92 seconds, 21.55 seconds, 21.34 seconds, 24.03 seconds, and 23.95 seconds, respectively. The average completion time of the six tasks by the proposed algorithm is 15.10 seconds, 15.00 seconds, 20.35 seconds, 20.60 seconds, 23.66 seconds, and 23.59 seconds. From the completion time point of view, the proposed virtual machine performance algorithm has shorter processing time and higher efficiency than genetic algorithm. In terms of stability, the genetic algorithm fluctuates greatly, so the proposed algorithm has higher stability.

In conclusion, in the prediction of spare parts demand with strong periodicity, the prediction method based on weighted fitting of eigenvalues has the smallest error and the optimal fitting effect in the prediction of machine spare parts demand, and the lowest error after fitting is only 2.2%. For spare parts with non-periodic linear demand and spare parts with nonlinear demand, exponential smoothing method and quadratic exponential smoothing method are used for prediction respectively, and the prediction results are close to the actual value. The spare parts demand prediction method proposed here can well complete the prediction for three different types of time series of demand data of spare parts, and the relative error of prediction is maintained at about 10%. The prediction effect can meet the basic requirements of spare parts demand prediction, and the prediction accuracy is higher than that of periodic prediction method. Compared with genetic algorithm, the cloud-edge collaborative computing algorithm for inventory management system takes less processing time and has higher efficiency. In terms of stability, genetic algorithm fluctuates greatly, but the algorithm reported here is much more stable.

## Conclusions

Efficient spare parts inventory management can reduce inventory costs, improve service level, and bring huge benefits to large equipment manufacturing enterprises. There are a variety of spare parts for large-scale equipment as well as many uncertain factors in the supply process. Therefore, it is essential to continuously update relevant technologies for higher efficiency of spare parts inventory management, to save inventory costs. Based on the supply chain background, the critical role of inventory management plan and spare parts demand relationship in improving the core competitiveness of enterprises. Secondly, according to different types of spare parts demand prediction data, different spare parts and demand prediction methods for vulnerable parts are proposed. In addition, the efficiency of inventory management is improved by predicting the demand for industrial vulnerable parts. For the three spare demand models of vulnerable parts, including periodic model, stationary model, and trend model, the corresponding demand forecasting methods are studied respectively. The simple exponential smoothing method is used to predict the spare parts with stable demands, while the quadratic exponential smoothing method is used to predict the demand for spare parts with linear trend. Meanwhile, the prediction method based on weighted fitting of eigenvalues is adopted to predict the periodical demand of machine spare parts. Finally, an inventory management system based on cloud-edge collaborative computing is proposed to reasonably allocate inventory resources and improve the utilization of inventory resources. The prediction method based on weighted fitting of eigenvalues proposed here has the smallest error and the best fitting effect in the demand prediction of machine spare parts, and the lowest error after fitting is only 2.2%. Exponential smoothing method and quadratic exponential smoothing method are used for spare parts with non-periodic linear demands and spare parts with nonlinear demands, respectively, and the prediction results are close to the actual values. In terms of completion time, the virtual machine performance algorithm reported here realizes shorter processing time and higher efficiency than genetic algorithm. In terms of stability, this research algorithm is much more stable than the genetic algorithm. Despite particular outcomes achieved in this work, due to the limitations of research level and some objective factors, there are still some deficiencies. On the one hand, there remains space for improvement in the relative error of the prediction method for vulnerable spare parts proposed here. It is expected to further improve the accuracy and efficiency of prediction by introducing the deep learning algorithm in future. On the other hand, there lacks the combination of the prediction method based on vulnerable spare parts and the inventory management system based on cloud-edge collaborative computing reported here. The follow-up work will make efforts to integrate spare parts demand forecasting and inventory resource management into one intelligent system.

## Supporting information

S1 Data (ZIP)
